RETRACTED

# A DSGE Decision Model for Investigating the LPR Transmission Effect

**DOI:** 10.1155/2022/2981558

**Published:** 2022-01-21

**Authors:** Xing Yang

**Affiliations:** School of Economics and Management, Beijing Jiaotong University, Beijing 100044, China

## Abstract

In August 2019, People's Bank of China launched the reform of Loan Prime Rate (LPR) quotation formation mechanism and then made continuous progress in the order of “new loans first, followed by exiting loans,” dredging the interest rate transmission channel of “policy interest rate, LPR, loan interest rate.” In 2020, Chinese financial institutions have mainly referred to LPR pricing for loans, and the marketization level of loan pricing has significantly improved. This paper analyzed the policy effects transmitted by LPR through constructing a Dynamic Stochastic General Equilibrium (DSGE) decision model, and it was found that the financial market structure, pricing ability of commercial banks, and the degree of LPR application all affected the policy rate transmission effect and had an impulse impact on macroeconomic growth. Based on the above analysis, this paper proposed policy suggestions on the path of interest rate market-oriented reform and coping measures of commercial banks in China.

## 1. Introduction

In August 2019, the market-oriented reform of China's interest rate was further deepened. People's Bank of China launched the reform of the formation mechanism of LPR in the loan market and continued to promote it in the order of “new loans first, followed by exiting loans,” forming a rate transmission mechanism of “policy interest rate, LPR, loan interest rate.” By the end of 2020, Chinese financial institutions have mainly referred to LPR pricing for loans, and the marketization level of loan pricing has significantly improved. However, it is worth noting that China's financial system structure is dominated by indirect financing, and there are some problems such as information asymmetry, implicit high leverage, and inadequate expectation management in the financial market. It is difficult to give full play to the profit-seeking function of capital, and the actual impact of interest rate reform on economic output is worth discussing. From the perspective of international experience, through the reform of interest rate marketization, it is conducive to narrowing the interest rate corridor, reducing short-term interest rate fluctuations, enhancing the sensitivity of real economic deposits interest rate and loan interest rate to policy interest rate, improving the transmission efficiency of monetary policy between different interest rates, and strengthening financial services in the real economy. Under the background of the imperfect system of China's financial market, after the reform of the LPR pricing mechanism, how efficient is the transmission efficiency of monetary policy? What is the actual impact on economic output? These are all issues that need to be studied. The study of the above problems will help us to further dredge the transmission path of monetary policy in a targeted manner, reduce the financing cost of the real economy, force the market-oriented development of the pricing method of funds of commercial banks, and further improve the efficiency of macroeconomic regulation and control.

RETRACTED

Therefore, it is of great significance to study the transmission effect of LPR pricing mechanism and its impact on economic growth. At present, the research mainly focuses on the effect evaluation of quantitative control tools and price control tools of monetary policy and the effect evaluation of interest rate regulation and interest rate market-oriented reform, and some studies believe that too fast interest rate market-oriented reform will increase the risk of financial institutions. However, there is a lack of research on the transmission effectiveness of LPR interest rate reform and the impulse impact on macroeconomic growth under different degrees of marketization. In order to further explore these questions, the paper constructs a DSGE model with financial market friction, studies the marketization degree in the process of LPR reform by difference scenarios, and analyzes the effectiveness of models such as calibration analysis, parameter estimation, and impulse response, so as to provide objective theoretical support for a comprehensive understanding of the policy effect of LPR.

## 2. Literature Review

The study on the transmission effect of monetary policy rate began as early as the late 19th century. Tobin [1] and Modigliani [2] pointed out that monetary policy transmission relied on not only interest rate transmission channels, but also nonmonetary assets price channels, such as enterprise Tobin's Q channel (assets price), the resident's wealth effect channel, and the exchange rate channel for transmission. Relying on the IS-LM model, Bernanke and Blinder [3] and Bernanke and Gertler [4] explained that not only the total money supply from the central bank, but also changes of bank credit supply quantity, both have a significant impact on monetary policy transmission. Due to incomplete information and agency costs in financial markets, expansion or shrinkage of bank credit quantity can cause economic agents to make different financing decisions and affect economic behaviors such as investment, consumption, etc. According to the above viewpoints, Mishkin [5] divide the monetary policy transmission channels into the interest channel, the credit channel, the assets price channel, and the exchange rate channel. Since then, a large number of empirical studies have begun to quantitatively measure the transmission efficiency of different channels. For example, Evans and Mashall [6] used Vector Autoregressive model (VAR) to study the role of monetary policy and inflation expectation on the term structure of interest rate and pointed out that tight monetary policy had a positive but temporary effect on short-term interest rate, while long-term interest rate was almost not affected. De Bondt [7] studied the European banking sector and found out through analysis that the market structure of the banking sector affected the transmission effect of monetary policy to some extent. The highly monopolistic banking would weaken the transmission effect of monetary policy, while market-oriented banking would make commercial banks more sensitive to interest rate changes and improve the transmission effect of the central bank monetary policy. Bolton and Freixas [8] further indicated that the capital adequacy ratio rules of commercial banks, while enhancing the risk prevention ability of commercial banks, reduced the ability of commercial banks to derivate money and weakened the transmission effect of the central bank's monetary policy in the commercial bank system. Milani and Treadwell [9] and Gomes et al. [10] show that the monetary policy with full expectation management has greater degree of macrocontrol on the economy and longer attenuation period of impact effect. Empirical studies on DSGE models based on open economy done by Meinusch and Tillmann [11] and Ge [12] manifest that the transmission efficiency of price monetary policy shows a significant improvement trend during the sample period, while the macrocontrol effect of quantitative monetary policy is gradually weakening.

RETRACTED

At present, the domestic literature on interest rate transmission mainly focuses on the transmission effect study of traditional loan and deposit benchmark rates, while there are few studies on transmission effect of LPR reform. Yingkun Jiang et al. [13] argued that the bank credit transmission channel played an important role in China's monetary policy transmission channels. However, the constraints of China's traditional credit system, as well as the state-owned nature and limited competition of commercial banks, can slow down the central bank's interest rate policy transmission and cause efficiency losses. Dong He and Honglin Wang [14] pointed out that, different from developed countries, China gradually formed a monetary policy framework with the dual interest rate system as the main feature in the market-oriented reform. China transmitted the monetary policy to market interest rate through various policy instruments and realized the monetary policy regulation with the credit quantity. Li Ma et al. [15] showed that the deposit reserve ratios of commercial banks were important factors that restricted the interest rate policy transmission effect of commercial banks. Deposit reserve ratio adjustment could guide market changes and macroeconomic development and promote the transmission effect of monetary policy by changing the adaptive expectations of market participants. Jun Ma et al. [16] constructed a DSGE decision model and pointed out that China's financial system, with indirect financing as the main body, faced many institutional constraints. The transmission of central bank's policy rate adjustment to each financial market rate would be influenced by China's financial market structure, loan scale restrictions, deposit reserve ratio, etc. Daoping Wang [17] used the panel data of 88 countries around the world to study the relationship between interest rate marketization and banking crisis which also shows that the improvement of marketization will significantly increase the probability of banking crisis. Ning Xu et al. [18] believed that China's LPR reform based on Medium-Term Lending Facility (MLF) tends to be more market-oriented and improves the transmission efficiency of monetary policy.

In summary, the existing research results showed that, due to China's monetary market structure with indirect financing as the main body, policy rate changes were mainly transmitted through bank credit. But the transmission mechanism was not smooth enough and the effectiveness of interest rate policy was low due to factors such as capital constraints of commercial banks, deposit reserve ratio constraints, and prudent management behaviors under imperfect competition. At present, the LPR interest rate has a typical market-oriented attribute, but its transmission efficiency and impact on economic growth are still lacking forward-looking empirical analysis. Based on the research methods of Zihan Huo et al. [19] and Long Zhang et al. [20] using DSGE model to analyze the impact effect of China's monetary policy on macroeconomy, this paper constructs a DSGE model including five subjects: government, residents, enterprises, central bank, and commercial banks to perspective dynamic changes of the regulation effect of LPR channel, in order to provide reference for improving the regulation of monetary policy.

## 3. Research Mechanism

### 3.1. Transmission Mechanism of Price-Based Regulatory Monetary Policy

When a country's economy is in a rising phase, the actual GDP growth rate is often higher than the country's potential economic growth rate, which tends to cause a continuous rise in CPI and drives residents' inflation expectations, thus intensifying the inflationary trend. To prevent the overheated economic fluctuations, the country's government often adopts a tight monetary policy to hold down the inflationary trend. In the price-based monetary policy regulation, the monetary authority often stimulates the rise in the financial market interest rate through open market operations, which makes medium- and long-term funds flow into the capital market. The shortage of funds will prompt commercial banks to increase the loan rate and squeeze the momentum of enterprise investment, raising the enterprise investment cost and slowing down the trend of overheated economy.

RETRACTED

When a country's economy is in a downward phase, the actual GDP growth rate is usually lower than the country's potential economic growth rate, resulting in a continuous downturn of the CPI and causing deflation. Therefore, it is required to implement an accommodative monetary policy to stimulate economic growth. In the price-based monetary policy regulation, the monetary authority often promotes the decline of financial market interest rate through open market operations to squeeze medium- and long-term capital outflows from the capital market. The sufficient funds will prompt commercial banks to reduce loan rate, which is conducive to enterprises to increase the investment scale, thus promoting economic recovery.

Since the mid-20th century, major developed countries have successively improved their monetary operation procedures by implementing a deposit and loan facility system, increasing the frequency of open market operations, narrowing the interest rate corridor range, as well as carrying out interest compensation on deposit reserves, adopting average reserve assessment, strengthening policy communication, and improving transparency, which can make money market interest rate deviate less from the central bank's target level and is more beneficial to the interest rate guidance of central bank. In October 2006, People's Bank of China introduced Shanghai overnight interbank offered rate (Shibor) by borrowing from London interbank offered rate (Libor), Euro interbank offered rate (Euribor), and other interest rates and made an active exploration in cultivating the market benchmark interest rate. However, due to the great fluctuation of Shibor in actual operation, combined with the single transaction structure of the money market, the borrowed funds basically showed a single flow direction (from large banks to small-sized and medium-sized banks), while large banks all belonged to the price quotation units of Shibor interest rate, which was easy to form a monopolistic interest rate to some extent, and had low market recognition as a monetary policy benchmark interest rate. In this process, People's Bank of China continuously enriched the means of interest rate regulation, built long-term, medium-term, and short-term policy interest rate system including 3-month, 6-month, and 1-year MLF interest rate and improved the efficiency of monetary policy interest rate transmission.

RETRACTED

### 3.2. Four Stages of LPR Mechanism Transmission

In October 2013, People's Bank of China launched the LPR, aiming to further stimulate market-oriented reform, improve the benchmark interest rate system, and guide the pricing of loan on credit market products. However, the LPR has been following the 1-year benchmark interest rate of loans announced by the central bank, and the interest rate level has been maintained at around 4.31%, which is much higher than the 1-year MLF interest rate of 3.30% and the 1-year Shibor interest rate of 3.52%. In August 2019, People's Bank of China further optimized the calculation method of LPR based on the mode of “new loans first, followed by exiting loans,” adopted the way of 1-year LPR equal to 1-year MLF plus base point for loans, and expanded the range of quoting banks. From the current operation condition, the transmission can be divided into four stages: In the first stage, the central bank lowers the MLF quotation rate to influence the financial market interest rate. In the second stage, the quoting bank adopts the way of “MLF + base point” for the LPR quotation, which should be calculated and published by China Interbank Offer Center. In the third stage, commercial banks adjust the loan rate according to the LPR quotation. In the fourth stage, commercial bank lending rate affects the investment and financing decisions and costs of enterprises and residents, thus affecting macrotargets such as economic growth, inflation, and employment. The transmission path is MLF⟶LPR⟶commercial bank lending rate⟶real economy⟶economic target (Figure 1).

In 2019, only 20% of the loans of Chinese commercial banks were floating priced up and down according to the LPR quotation, and about 80% of the loans were still floating priced up and down according to the loan benchmark interest rate published by the central bank in the past. By the end of 2020, commercial bank loans had realized transformation from policy benchmark interest rate to market interest rate, so as to ensure that the policy operation intention of People's Bank of China can be effectively transmitted to other markets.

RETRACTED

### 3.3. Main Idea of DSGE Decision Model Construction

The estimation of the DSGE decision model is generally divided into three steps: First, based on the economics theory and the economic operation characteristics in China, the optimal behavior characteristic of each economic agent when the economic system is in equilibrium is set. Second, the policy equation of the economic variables is solved, and the model parameters are estimated by running calibration and Bayesian estimation. Third, the impulse response is used to carry out efficiency analysis of the model and test the explanatory ability of the model for the actual economic problems.

Foreign studies on the transmission mechanism of monetary policy mainly focus on how market rate changes affect economic operation through financial markets, while there are few studies on the impact of policy rate changes transmitted to the real economy. This is mainly because the financial systems of developed countries are often dominated by the direct financing market, where regulatory policies have fewer constraints on financial markets and benchmark market interest rate is mostly determined by transactions between financial markets. In contrast, China's financial system is dominated by the indirect financing market, where the policy rate changes have a significant impact on the real economy. Based on this, this paper constructs a DSGE model that includes five entities: government, residents, enterprises, central banks, and commercial banks, and defines the corporate loan interest rate as adjusting according to the LPR pricing level and according to the three scenarios of 50%, 80%, and 100% loans with reference to LPR pricing, to discuss the impact of the change of the unit policy interest rate on economic growth.

## 4. Research Method

### 4.1. DSGE Decision Model Frameworks of 5 Sectors

#### 4.1.1. Resident Sector

The resident sector realizes the maximization of economic utility by supplying labor, earning income, and consumption. Its utility equation is as follows:

(1) $$\begin{array}{c} U\left(C_{t},N_{t},\frac{M_{t}}{P_{t}}\right)=Z_{t}^{c}\frac{C_{t}^{1-\sigma_{c}}}{1-\sigma_{c}}+Z_{t}^{m}\frac{{\left(M_{t}/P_{t}\right)}^{1-\sigma_{m}}}{1-\sigma_{m}}-Z_{t}^{n}\frac{N_{t}^{1+\sigma_{n}}}{1+\sigma_{n}}. \end{array}$$

The expected utility is

(2) $$\begin{array}{c} \text{max}:E_{t}\left[\sum_{t=0}^{\infty }\beta^{t}U\left(C_{t},N_{t},\frac{M_{t}}{P_{t}}\right)\right]. \end{array}$$

The constraint condition is

(3) $$\begin{array}{c} \text{s}.\text{t}:C_{t}+\frac{M_{t}}{P_{t}}=\alpha_{t}^{s}N_{t}^{s}+\frac{M_{t-1}}{P_{t}}, \end{array}$$

where *E*_*t*_ is the mathematical expectation, and *β*^*t*^ is the discount factor (0 < *β* ≤ 1). *C*_*t*_ is the household consumption level, and *N*_*t*_ is the labor supply of the household to society. *M*_*t*_ is the nominal assets balance held by the household, and *P*_*t*_ is the product price in the current period. *M*_*t*−1_ is the household's nominal assets balance held in period t-1 and substituted into period *t*. (*M*_*t*_/*P*_*t*_) is the actual assets balance held by the household. *Z*_*t*_^*c*^, *Z*_*t*_^*m*^, and *Z*_*t*_^*n*^ are exogenous impact variables for consumption demand, labor supply, and holding assets, respectively. *σ*_*c*_, *σ*_*n*_, and *σ*_*m*_ are the consumption demand elasticity, labor supply elasticity, and money demand elasticity, respectively. *α*_*t*_^*s*^ is the average wage level.

RETRACTED

#### 4.1.2. Enterprise Sector

The enterprise sector obtains the maximum enterprise welfare by investing capital and labor. The objective function is max : *E*_*t*_[∑_*t*=0_^*∞*^*β*_*t*_^*p*^ lg*C*_*t*_^*p*^] , where *β*_*t*_^*p*^ is the discount rate of the manufacturer and *C*_*t*_^*p*^ is the remuneration obtained by the business owner. Suppose the production equation of the manufacturer is

(4) $$\begin{array}{c} Y_{t}^{p}=A_{t}^{P}{\left(K_{t}^{p}\right)}^{\alpha_{1}}{\left(N_{t}^{p}\right)}^{1-\alpha_{1}}, \end{array}$$

where *Y*_*t*_^*p*^ is the output of the enterprise, and *A*_*t*_^*P*^ is the production technology level of the enterprise. *K*_*t*_^*p*^ is the capital invested by the enterprise, and *N*_*t*_^*p*^ is the labor invested by the enterprise. *α*_1_ is the output elasticity of capital input, and *α*_1_*ϵ*(0,  1).

Refer to the research of Xiangyang Li et al. [21]; this paper assumes that the resource constraint equations of the enterprise are as follows:

(5) $$\begin{array}{c} \left(1-T_{p}\right)Y_{t}^{p}+L_{t}^{p}+\left(1-\varepsilon \right)K_{t-1}^{P}-L_{t-1}^{p}\frac{1+R_{t}^{p}}{\pi_{t}},\\ C_{r}^{p}-K_{t}^{p}=0,\\ L_{t}^{p}\frac{1+R_{t}^{p}}{\pi_{t}}=m_{p}K_{t}^{p}, \end{array}$$

where *T*_*p*_ is the tax rate to be paid by the enterprise, and *ε* is the depreciation rate. *L*_*t*_^*p*^ is the loan balance obtained by the enterprise in period *t*, and *R*_*t*_^*p*^ is the loan interest rate. *m*_*p*_ is the asset-liability ratio of the enterprise. Enterprise loans are generally restricted by the loan interest rate and the asset-liability ratio.

#### 4.1.3. Government Sector

The basic behavior characteristics of the government are simply simulated in this model; that is, the government obtains funds through tax revenue and debts, and these funds are mainly used for government investment and government consumption, except for paying back debt and interest of the last period. The government budget constraint is

(6) $$\begin{array}{c} \frac{g_{t}}{p_{t}}+T_{t}+T_{p}Y^{t}=B_{t}+G_{t}, \end{array}$$

where *g*_*t*_ is the funds received by the government from issuing treasury bonds, and *P*_*t*_ is the inflationary price of the current period. *T*_*t*_ is the tax revenue paid by the residents and *T*_*p*_*Y*^*t*^ is the government tax revenue (where *T*_*p*_ is the tax rate and *Y*^*t*^ is the enterprise output). *B*_*t*_ is the government consumption expenditure, and *G*_*t*_ is the government investment expenditure.

RETRACTED

#### 4.1.4. Central Bank

People's Bank of China is now gradually abandoning the money supply as the intermediate target and more focusing on the adoption of policy rate. There are generally 4 ultimate objectives: price stability, promoting economic growth, maintaining employment, and balance of international payment. However, considering Mundell's Impossible Trinity, this paper mainly considered price stability, economic growth, and maintaining employment. Accordingly, the monetary policy constraint equation of People's Bank of China is as follows:

(7) $$\begin{array}{c} \frac{R_{t}}{R}={\left(\frac{Rt}{R_{t-1}}\right)}^{\theta_{R}}{\left[{\left(\frac{\pi_{t}}{\pi_{t-1}}\right)}^{\varphi_{\pi }}{\left(\frac{Y_{t}}{Y_{t-1}}\right)}^{\varphi_{y}}{\left(\frac{M_{t}}{M_{t-1}}\right)}^{\varphi_{m}}{\left(\frac{p_{t}}{p_{t-1}}\right)}^{\varphi_{p}}\right]}^{1-\theta_{R}}{Ζ}_{\iota }^{r}, \end{array}$$

where (*Rt*/*R*_*t*−1_) is the changing value of policy rate (this paper adopted MLF interest rate). (*M*_*t*_/*M*_*t*−1_) is the changing value of money supply and (*π*_*t*_/*π*_*t*−1_) is the changing value of unemployment rate. (*Y*_*t*_/*Y*_*t*−1_) is the changing value of total social output, and (*p*_*t*_/*p*_*t*−1_) is the changing value of inflation rate. The parameters *θ*_*R*_, *φ*_*π*_, *φ*_*y*_, *φ*_*m*_, and *φ*_*p*_ are the elasticity of interest rate, unemployment rate, total output, money supply, and inflation from their steady-state deviation degree with respect to interest rate, respectively. Ζ_*ι*_^*r*^ is the exogenous impact variable of China's monetary policy.

#### 4.1.5. Commercial Bank

Commercial banks mainly face Net Interest Margin (NIM) constraints in business operations. Commercial banks earn interest income from loans to cover the deposit interest cost and maintain interest spread income. Therefore, the budget constraint equation for commercial banks is as follows:

(8) $$\begin{array}{c} D_{t}r_{t}+F_{t}=L_{t}^{p}R_{t}^{p}+B_{t}^{G}R_{t}^{G},\\ R_{t}^{p}=LPR_{t}+K_{t}, \end{array}$$

where *r*_*t*_ is the deposit interest rate, and *D*_*t*_ is the commercial bank deposit balance. *F*_*t*_ is the commercial bank profit, and *R*_*t*_^*p*^ is the enterprise loan interest rate (LPR_*t*_ plus floating point *K*_*t*_). *R*_*t*_^*G*^ is the government financing rate. *L*_*t*_^*p*^ is the balance of enterprise loans and *B*_*t*_^*G*^ is the balance of government financing.

RETRACTED

### 4.2. Data Selection, Parameter Calibration, and Economic Steady State

We consider that *Y*=*C*_*t*_+*Y*_*t*_+*F*_*t*_+*G*_*t*_+*R*_*t*_. Among them, Y represents the total output of the economy, *C*_*t*_ represents the resident sector, *Y*_*t*_ represents the corporate sector, *B*_*t*_ represents the commercial banking sector, *G*_*t*_ represents the government sector, and *R*_*t*_  represents the central bank sector. In order to further examine the effectiveness and efficiency of monetary policy transmission after the implementation of LPR reform, we will select the main observation data according to the DSGE model framework of the five departments and simulate the transmission of monetary policy by means of calibration analysis.

#### 4.2.1. Data Selection

The sample interval for this section is from January 1980 to December 2021. The main observational variables include interest rate data (1-year MLF interest rate, 1-year LPR interest rate, 1-year bank deposit rate, 1-year bank loan interest rate, and 1-year treasury bond interest rate); bank data (bank deposit balance as a proportion of GDP, bank loan balance as a proportion of GDP, new loans to new social financing, new government bonds to new social financing, and bank net interest margin); economic data (GDP growth rate, inflation rate, unemployment rate, M2 growth rate, and corporate asset-liability ratio). The data are all from the WIND database. Here, considering the substitution of wealth management products for resident deposits, the deposit interest rate adopts the average expected yield of 1-year wealth management products of large commercial banks. This paper first deflates GDP, bank deposits, and bank loans, then uses the X12 method to seasonally adjust all data, and finally takes all the data logarithmic and first-order differences. The statistical description of the data is shown in Table 1.

#### 4.2.2. Parameter Calibration

The steady-state value of the variable *R*_*t*_ is defined as *R*_*t*_^*∗*^, and $\hat{{\text{R}}_{t}}$ is the steady-state deviation of the variable *R*_*t*_ with respect to *R*_*t*_^*∗*^, that is, $\hat{R_{t}}=\log\;R_{t}-\log\;R_{t}^{*}$. The linear policy equation of the DSGE decision model can be obtained by conducting first-order differential and first-order Taylor expansion. After that, the a priori calibration method and automatic model solution are required to obtain the estimated values of the parameters.

RETRACTED

In this paper, Carlstrom et al. [22] study and calibrate some static parameters with relatively stable values and then focus on the Bayes method to estimate the dynamic structural parameters related to the degree of marketization and interest rate transmission. For example, this article uses *θ*_*R*_ as an indicator of the degree of financialization; we estimated three marketization degree coefficients based on three samples of different periods, of which from January 1980 to December 2007, the marketization degree coefficient was 0.012, which was the interest rate control stage; from January 2008 to December 2018, the marketization degree coefficient was 0.4523, and the market benchmark interest rate system represented by Shibor was constructed, which was the market cultivation stage; from January 2019 to December 2021, with the advancement of the reform of China's LPR interest rate pricing system, the degree of marketization coefficient was 0.6851, which was the stage of gradual market liberalization. Considering the above factors, the final calibration value of *θ*_*R*_ is 0.4832. The estimation results are shown in Table 2.

#### 4.2.3. Steady-State Simulation

This section uses the impulse response analysis of the DSGE model to explore the role of changes in the benchmark interest rate of monetary policy on economic output. When People's Bank of China lowers the MLF rate, the LPR goes down and affects the total output of the economy through the response of banks, businesses, and residents and then gradually returns to the vicinity of steady state. Taking into account the uncertainty of COVID-19 in 2020–2021, this is a comparative analysis of the 2019 national economic statistics before the epidemic: in the year LPR (1 year) dropped 3 times, with a year-end value of 4.15%, which was down by 26BP compared with the beginning of the year. The LPR (5-year period) was set up in August 2019, 1 time lower, and the value at the end of the year was 4.80%, which decreased by 5BP compared with the initial value. The annual price index is 102.90%, with an increase of 0.2 percentage point from the previous year. The proportion of RMB loans balance as a percentage of GDP is 154.52% and the proportion of RMB deposit balance as a percentage of GDP is 97.10%. The new RMB loans account for 66.0% of the new social financing scale in the same year. The year-on-year growth rate of the money supply M2 balance is 8.70%, with an increase of 0.1 percentage point from the previous year. The NIM of commercial banks is 2.19%, with an increase of 0.14 percentage point compared with the end of the previous year (Table 3).

RETRACTED

This paper analyzes the matching degree between benchmark model simulation results and China's macroeconomic data in 2019 in terms of interest rate level, bank scale, and the real economy.

In terms of policy rate level, the 1-year MLF interest rate (3.35%) and LPR interest rate (4.90%) simulated by the model are both higher than the corresponding actual interest rate levels. The simulated loan interest rate (5.25%), deposit interest rate (2.80%), and government bond interest rate (2.70%) are all lower than the corresponding actual interest rate levels. This indicates that the monetary policy transmission mechanism in China still has a serious obstacle in practice. The prudent risk behavior of the banking system in the credit process makes its loans with a relatively long period and large loan limit and concentration; i.e., the actual loan interest rate corresponding to the policy rate is higher than the equilibrium interest rate level simulated by the model. The actual deposit interest rate corresponding to the policy rate is also higher than the equilibrium interest rate simulated by the model due to the competition for residents' deposits and the substitution of fixed time and current deposits by certificate deposits and finance products.

In terms of bank scale, the proportions of deposit and loan balances as a percentage of GDP simulated by the model are highly consistent with the actual data. However, the proportion of new loans as a percentage of new social financing is lower than the actual value, and the proportion of new government bonds as a percentage of new social financing is higher than the actual value, which indicates that China's financial market structure is still unsatisfactory, with a high proportion of credit financing and a relatively low proportion of capital market financing. The net interest margin enjoyed by Chinese commercial banks is still higher than the equilibrium value due to the blockage of policy rate transmission, indicating that the policy dividends still exist.

In terms of the development of the real economy, the GDP growth rate, inflation rate, unemployment rate, M2 growth rate, and enterprise asset-liability ratio simulated by the model are all superior to the actual data, which indicates that the blockage of policy rate transmission has aggravated the business difficulties of the real economy and reduced the operating efficiency of China's economy.

## 5. Results and Discussion

This paper used the Dynare tool to estimate the dynamic response of each variable in the economy to the temporary impact of the given policy rate with the advancement of the LPR interest rate reform. Specifically, it can be divided into the following scenarios: (i) LPR pricing mechanism loans account for 50% of the existing loans; (ii) LPR pricing mechanism loans account for 80% of the existing loans; (iii) LPR pricing mechanism loans account for 100% of the existing loans. This paper takes the weighted average interest rate of one-year loan, the interest rate of one-year time deposit, and the yield of one-year treasury bond as observation variables.

RETRACTED

From August 2019 to the end of 2021, in order to hedge the impact of COVID-19, China's monetary policy was in an easing cycle. The 1-year LPR interest rate has been lowered by 6 times and the cumulative 35BP has been lowered.

### 5.1. LPR Pricing Mechanism Loans Account for 50% of the Exiting Loans

In this scenario, we assume that there are no other changes in policy constraints. The model results showed that when the policy rate decreased by 35 BP, the loan interest rate, deposit interest rate, and government bond interest rate declined by 21 BP, 15 BP, and 26 BP. This indicates that when LPR pricing mechanism loans account for 50% of the existing loans, the transmission efficiencies of the policy rate to the loan interest rate, deposit interest rate, and government bond interest rate are 60%, 43%, and 74%, respectively (Figure 2).

Generally speaking, when the policy rate falls, the price of borrowing funds from the central bank by commercial banks decreases, and commercial banks will reduce their demand for deposits, thus resulting in a decline in deposit interest rate, which in turn leads to a diversion of residents' deposits to Internet finance as well as the stock and bond markets. In practice, however, the falling range of deposit interest rate will be smaller because the deposit interest rate is relatively stable, while commercial banks, due to the price reduction of funding sources, will cut enterprise loan interest rate accordingly in order to gain more loan market shares, thus bringing down the enterprise financing cost. Accordingly, the price of bond financing in the financial market will also decline. Therefore, from the model, when the policy rate decreases, the loan scale of commercial banks will increase, while the deposit scale will decline.

### 5.2. LPR Pricing Mechanism Loans Account for 80% of the Exiting Loans

Similarly, in this scenario, we assume that there are no other changes in policy constraints. The model results showed that when the policy rate decreased by 35 BP, the loan interest rate, deposit interest rate, and government bond interest rate declined by 24 BP, 18 BP, and 29 BP, respectively. Thus it is indicated that when LPR pricing mechanism loans account for 80% of the existing loans, the transmission efficiencies of the policy rate to the loan interest rate, deposit interest rate, and policy bond interest rate are 69%, 51%, and 83%, respectively.

RETRACTED

### 5.3. When LPR Pricing Mechanism Loans Account for 100% of the Existing Loans, The Benchmark Interest Rates of Deposits and Loans Are Removed

Similarly, in this scenario, we assume that there are no other changes in policy constraints. The model results showed that when the policy rate decreased by 35 BP, the loan interest rate, deposit interest rate, and government bond interest rate declined by 28 BP, 25 BP, and 32 BP, respectively. Thus it is indicated that when LPR pricing mechanism loans account for 100% of the existing loans, the transmission efficiencies of the policy rate to the loan interest rate, deposit interest rate, and policy bond interest rate are 80%, 71%, and 91%, respectively.

### 5.4. The Impact Effect of a Unit Interest Rate Change on Economic Output under Three Different Scenarios

Under the above three different marketization degrees, the adjustment of LPR interest rate can have an impact on the actual output. Further observing the impulse intensity under different marketization degrees, we can find that, with the continuous relaxation of interest rate control, output is becoming more sensitive to interest rate adjustments. From the perspective of transmission mechanism, the reduction of LPR interest rate means the decline of policy interest rate, which is a loose monetary policy and can effectively promote economic growth. This paper uses the year-on-year growth of real GDP as the measurement index of economic output and uses Dynare tool to estimate the impact of economic output on the temporary impact of reducing one unit of LPR interest rate. The following results can be obtained: during the period when the LPR pricing mechanism loans account for 50% of the loan stock, reducing the LPR interest rate by 1 BP will increase the year-on-year growth rate of real GDP by 0.005 percentage points; in the period when the LPR pricing mechanism loan accounts for 80% of the loan stock, reducing the LPR interest rate by 1 BP will increase the year-on-year growth rate of real GDP by 0.009 percentage points; in the period when the LPR pricing mechanism loan accounts for 100% of the loan stock, reducing the LPR interest rate by 1 BP will increase the year-on-year growth rate of real GDP by 0.012 percentage points, as shown in Figure 3.

The results show that the LPR pricing system reform implemented by People's Bank of China makes the interest rate marketization enter a new stage, can effectively improve the interest rate transmission efficiency of monetary policy, and plays a positive role in promoting economic growth. First, it really decouples the loan pricing of commercial banks from the policy benchmark interest rate and promotes the LPR interest rate to 100% existing loan pricing, indicating the substantive progress in the market-oriented reform of interest rate; second, it adopts the gradual principle to promote the application of LPR interest rate and takes MLF interest rate as the reference standard to prevent the excessive fluctuation of market interest rate to a certain extent; third, LPR interest rate has a certain impact on real GDP growth, and the impact effects are quite different under different marketization degrees, which means that financial market friction has a certain obstacle to the transmission efficiency of monetary policy. Since LPR not only inherits the advantages of gradual reform, but also integrates market-oriented elements, the interest rate transmission mechanism after its emergence needs to be researched. In addition, it is worth noting that the monetary transmission efficiency in the DSGE theoretical model is generally better than the actual data. This means that the efficiency loss faced by monetary policy in the actual transmission process during the regulation period is much greater than the theoretical expectation. At the same time, it also shows that LPR, an important reform that takes into account both robustness and market attributes, will become a useful attempt in the process of interest rate marketization.

RETRACTED

## 6. Research Conclusions

This paper constructs a DSGE model to compare and analyze the impact of LPR reform on monetary policy transmission mechanism and economic output under different marketization degrees and mainly draws the following conclusions. First, interest rate regulation has a real loss on the transmission efficiency of monetary policy, which is far greater than the theoretical expectation; second, with the advance of LPR reform, the response of real GDP year-on-year growth to LPR interest rate has become more and more sensitive, indicating that LPR interest rate reform can effectively affect economic growth; third, the higher the degree of marketization of LPR interest rate is, the more significant the transmission effect on deposit interest rate, loan interest rate, and treasury bond interest rate will be, and the efficiency of interest rate transmission mechanism will be improved. Consider that LPR pricing mechanism is still in the process of improvement, and in the meantime, there is a negative impact of COVID-19 on China's economy. The empirical results of this paper need to be further improved and verified.

RETRACTED

At the same time, we still need to deeply realize that there are still some differences between the theoretical expectation and practical effect of the reform. Especially in the stage of complete marketization, the actual efficiency loss of progressive reform is much higher than the theoretical expectation. For example, at the beginning of implementing the interest rate corridor model by the European Central Bank, the width of the interest rate corridor reached 250 BP. After 2003, in the face of the chain impact of the subprime mortgage crisis of the US, the European Central Bank continuously narrowed the interest rate corridor, of which the interest rate corridor was narrowed to 100 BP in December 2008 and 50 BP in June 2014 and is now maintained at 65 BP. This has led to a sharp narrowing of the interest spreads of deposit and loan of commercial banks, and some banks have thus got into trouble. This means that there are many hidden costs in the regulated interest rate transmission mechanism. At the same time, it also shows that only by fundamentally promoting the complete market-oriented reform will the interest rate transmission efficiency be fundamentally changed.

It is suggested that People's Bank of China continues to strengthen its research on improving the marketization of interest rates: First, a more complete interest rate corridor mechanism should be created, and the interest rate corridor range should be gradually narrowed, so as to ensure to give full play the role of the interest rate corridor mechanism. Second, the monetary policy transmission mechanism should be improved, and the function of the MLF as a medium-term policy rate should be exerted while strengthening the guidance of short-term policy rate. Third, the benchmark interest rates of loans and deposits determined by the central bank should be removed appropriately. Fourth, the direct financing channels should be vigorously developed and the monetary policy transmission mechanism should be improved. In this process, as the LPR reform is a gradual implementation process, the depth and breadth of its application have an important impact on the transmission of policy rate to market rate.

It is suggested that the commercial banks actively adapt to the process of interest rate marketization reform. First, it is necessary to establish a more scientific and reasonable pricing mechanism and improve the depth of application of LPR. Second, it is necessary to enhance the foresight of interest rate risk management, establish a mechanism for hedging interest rate exposures, and reasonably use interest rate swaps and other derivative instruments to carry out hedging operations. Thirdly, the innovation of interest rate derivative products can ensure the effect of interest rate market reform and further unblock the efficiency of monetary policy transmission.

RETRACTED

## Figures and Tables

**Figure 1:** LPR mechanism transmission framework diagram.

**Figure 2:** Effect of LPR interest rate on deposit, loan, and treasury bond interest rate.

**Figure 3:** Impulse effect of LPR interest rate on economic growth under different degrees of marketization.

**Table 1:** Descriptive statistics of all variables.

Name	Obs	Mean	Std.	Min	Max

MLF interest rate	504	3.1341	0.5999	2.9500	3.3000
LPR interest rate	504	4.6842	1.7160	3.8000	5.7700
Deposit rate	504	4.9905	0.1464	3.000	30.0000
Loan interest rate	504	5.5948	0.8816	4.7500	7.5600
Treasury interest rates	504	2.6672	0.6976	0.8871	4.2503
Deposit balance/GDP	504	1.9433	0.2194	1.4102	2.3352
Loan balance/GDP	504	1.3778	0.2371	0.9579	1.9156
New loans/new social financing	504	0.6549	11.4001	0.4213	1.1563
New government bonds/new social financing	504	0.1143	6.7104	0.0171	0.2392
Bank NIM	504	2.3617	0.2622	2.0300	2.7700
GDP growth	504	0.1173	0.1026	0.0220	0.1423
CPI	504	2.6350	1.9774	−1.8000	8.7000
Jobless rate	504	4.0165	0.1647	3.6100	4.3000
M2 growth	504	13.0246	5.0742	8.0000	29.7400
Asset-liability ratio of industrial enterprises	504	0.6103	2.0045	0.5830	0.6420

**Table 2:** Calibration values of main parameters.

Interest rate level	Value	Parameter	Value	Parameter	Value

*β* ^*t*^	0.988	*T*_*p*_	0.412	*φ*_*π*_	0.023
*σ*_*c*_	0.331	*ε*	0.201	*φ*_*y*_	0.921
*σ*_*n*_	0.355	*β*_*t*_^*p*^	0.122	*φ*_*m*_	0.634
*σ*_*m*_	0.423	*r*_*t*_	0.311	*φ*_*p*_	0.123
*α*_1_	0.562	*θ*_*R*_	0.483	*m*_*p*_	0.913

**Table 3:** Comparison of model simulation results with actual data of China's economy (2019).

Interest rate level	*R*_*t*_	LPR_*t*_	*R*_*t*_^*p*^	*r*_*t*_	*R*_*t*_^*G*^

Model	3.35	4.90	5.25	2.80	2.70
Data	3.26	4.80	5.50	3.80	2.85
Bank scale	Deposit/GDP	Loans/GDP	New loans/new social financing	New government bonds/new social financing	Net interest margin
Model	96.7%	155.1%	60%	20%	2.05%
Data	97.1%	154.5%	66%	18.5%	2.19%
Real economy	GDP growth rate	Inflation rate	Unemployment rate	M2 growth rate	Enterprise asset-liability ratio
Model	6.3%	2.7%	4.3%	8.6%	62%
Data	6.1%	2.9%	4.5%	8.7%	64%

## Data Availability

The data were taken from the WIND database and relevant information from People's Bank of China. Due to confidentiality requirements, they cannot be provided to research institutions outside of mainland China.
